# Toward Sustainable Development: Unleashing the Mechanism Among International Technology Spillover, Institutional Quality, and Green Innovation Capability

This article has been retracted.

**DOI:** 10.3389/fpsyg.2022.912355

**Published:** 2022-07-29

**Authors:** Tao Wang, Yuan Ding, Ke Gao, Ruiqi Sun, Chen Wen, Bingzheng Yan

**Affiliations:** ^1^School of Public Finance and Taxation, Capital University of Economics and Business, Beijing, China; ^2^School of Management, Ocean University of China, Qingdao, China; ^3^Development Research Center of Shandong Provincial People’s Government, Jinan, China; ^4^School of Economics, Peking University, Beijing, China; ^5^The Center for Economic Research, Shandong University, Jinan, China; ^6^School of Finance, Renmin University of China, Beijing, China; ^7^School of Social Development and Public Policy, Fudan University, Shanghai, China

**Keywords:** international technology spillover, institutional quality, green innovation ability, interaction effect, dynamic threshold model

## Abstract

Under the background of sustainable development, China’s economic growth engine becomes innovation-driven, and it is an important way for China to rapidly improve its green innovation capability by opening up to the outside world and utilizing the spillover effect of international technology. In this article, the system quality evaluation system is reconstructed by the method of fully arranged polygonal graphical indicators, and the provincial system quality in China is measured and added into the model as a regulating variable. The dynamic panel method and the dynamic threshold panel method are used to test the direct effects of foreign direct investment (FDI) and foreign trade on green innovation capability, the interaction effect of institutional quality, and the threshold effect. Empirical results show that the three technology spillovers have significantly promoted China’s green innovation capability. System quality will affect the determining coefficient of international technology spillovers on China’s green innovation capability. The positive promoting effects of FDI and foreign trade on China’s green innovation capability, all increase with the improvement of China’s system quality. Therefore, when utilizing FDI and foreign trade to promote green innovation in each region, each region should consider creating a good institutional environment for the emergence of international technological effects.

## Introduction

After China’s economic development has entered a new normal, it is necessary to promote sustainable economic development (Ahmad et al., 2021; Yang et al., 2021; Fang et al., 2022) with green innovation (Wu et al., 2019; Zhu et al., 2019; Irfan et al., 2020). The report of the 19th National Congress of the Communist Party of China also emphasized many times that “innovation is the first driving force for development,” and technological innovation and scientific and technological progress play an important role in driving national economic development (Hao et al., 2021b). Despite the rapid development of China’s high-tech industry in recent years, the large investment in research and development (R&D) funds has not completely solved the problems of low efficiency of scientific and technological innovation and weak original innovation ability (Jinru et al., 2021; Irfan and Ahmad, 2022; Abbasi et al., 2022). The long-term existence of this phenomenon will definitely restrict the effective implementation of China’s green innovation-driven development strategy (Tang et al., 2021; Wu et al., 2021; Yan et al., 2021). China, as a developing country with a relatively backward technology level, started to implement the independent innovation strategy late (Rauf et al., 2021; Shao et al., 2021; Yumei et al., 2022), but it is still at the low end of the vertical division system of the global value chain (Elavarasan et al., 2021a,b; Tanveer et al., 2021). Nowadays, with the deepening of economic globalization, to make China an innovative country in 2035, it is an important way for China to rapidly improve its independent innovation capability to realize the spillover effect of international technology through the opening to the outside world (Hao et al., 2021a). Besides, whether international technology spillover can play its role smoothly and effectively, the key lies in the influence of the exogenous institutional environment, that is, institutional quality (Gokmenoglu et al., 2015; Hao et al., 2021b). Especially under the condition of an open economy, with the increase in production and transaction links that multinational corporations need to coordinate, if the transaction cost is too high and the transaction risk is difficult to control, it will inevitably hinder the emergence of an international technology spillover effect (Hao et al., 2020). Therefore, how to build a regional institutional quality environment with coordinated development of politics, economy, and law, and make the international technology spillover play the most effective role in improving the green innovation capability, has become an important issue in the development of China’s regional innovation capability.

At present, the research on how international technology spillovers affect green innovation capability has not reached a unanimous conclusion, and the absorption effect of international technology spillovers varies greatly in different countries and regions. Some scholars have pointed out that the reverse technology spillover of foreign trade or outward foreign direct investment (OFDI) can significantly enhance the regional innovation capability (Grossman and Helpman, 1993; Coe and Helpman, 1995; Lichtenberg and De La Potterie, 1998; Ho et al., 2013; Kim et al., 2016); while some scholars stressed that FDI or OFDI did not play a substantial role in promoting regional innovation capability (Bitzer and Kerekes, 2008). In addition, some scholars believe that the relationship between international technology spillover and the promotion of green innovation ability of the host country is not simply linear, which requires not only considering the type of foreign investment, it is also necessary to consider the host country’s human capital reserve, intellectual property protection, industrial structure, opening level, and other factors (Djankov and Hoekman, 2000; Uotila et al., 2005). Nelson, an American scholar, pointed out in the article “American System Supporting Progress” that reasonable institutional arrangements mainly consist of the market mechanism, intellectual property protection policy, and government role, and deeply analyzed that the innovation ability of the United States benefits from a high-quality social system. In fact, as the basic rule of social and economic operation, it has a profound impact on social development. Poor system quality will increase the tax burden of economic activities, increase transaction costs, and reduce operational efficiency. Problems, such as the administrative monopoly of local governments will also breed rent-seeking and corruption. Good system quality can not only reduce unnecessary obstacles, reduce transaction costs, and the breeding of corrupt rent-seeking activities, it can also reduce the uncertainty in the process of innovation and research, and promote the research, development, innovation, and application of advanced technologies (Shleifer, 1998; Huang and Xu, 1999; Falvey et al., 2006; Tebaldi and Elmslie, 2013). If an institutional system is established in the production activities of enterprises, which can not only effectively motivate people to engage in productive activities but also ensure that all parties involved can fairly realize their rights and obligations, it will not only help to improve the innovation ability but also promote the growth of economic performance of enterprises. Therefore, improving the system quality and creating conditions for the introduction and internalization of international advanced technology are the key to promoting the domestic green innovation capability by using international technology spillover.

Throughout the existing research, it is found that: (1) in the related research on the impact of international technology spillover on green innovation capability, there is a lack of systematic analysis from the perspective of institutional quality, and the selection of indicators is too single to fully reflect the connotation of institutional quality; (2) FDI, OFDI, or a single index of foreign trade are mostly used to measure the international technology spillover index, and few scholars put the three into the same framework for comprehensive consideration; and (3) most of them are limited to static analysis, and its potential endogenous problems will lead to estimation errors. Different from previous studies, this article combines the provincial panel data from 2010 to 2019 and adopts the method of fully arranged polygon graphic indicators to establish the regional system quality evaluation system (Ren et al., 2022). Using direct effect, interactive effect, and threshold effect, this article examines the relationship among international technology spillover, institutional quality, and green innovation capability, and systematically analyzes the influence mechanism of international technology spillover on green innovation capability. To provide theoretical and policy references for China to effectively utilize the spillover effect of international technology to enhance its green innovation capability and realize the transformation of its growth engine to an innovation drive as soon as possible.

## The Measurement and Analysis of System Quality

### Construction of a System Quality Index System

The institution quality is a rather broad concept. As pointed out by North (1989), institution quality should cover all aspects, such as law, property rights, government efficiency, and execution. Since 1978, the internal reform and opening-up to the outside world have undoubtedly been the periods when the quality of China’s system has changed most drastically. Under the dual background of internal system transformation and external economic impact, we need to use scientific evaluation methods to measure the system quality of provinces and regions in China. For the measurement of domestic institutional quality in China, its quantification is often subjective and difficult to measure. Therefore, following the research of Ren et al. (2021), this article takes the connotation of system quality as the guiding principle. Based on previous studies, the comprehensive evaluation system of system quality, including political, economical, and legal environment, is reconstructed (as shown in Table 1).

**TABLE 1:** Construction of a system quality index system.

Primary index	Secondary index	Three-level index	Four-level index	Index attribute
System quality	Legal system environment	Judicial protection level	Proportion of regional lawyers (*X_1_*)	Ascending type
		Administrative protection level	The settlement rate of patent infringement cases (*X_2_*)	Ascending type
			Case closing rate of counterfeiting others’ patents (*X_3_*)	Ascending type
		Level of economic development	Per capita GDP (*X_4_*)	Ascending type
		Educational development level	Proportion of junior college or above (*X_5_*)	Ascending type
			Proportion of high school education (*X_6_*)	Ascending type
			Proportion of junior high school education (*X_7_*)	Ascending type
			Proportion of primary schools (*X_8_*)	Ascending type
	Political environment	Regional corruption	The proportion of corrupt people involved (*X_9_*)	Constraint type
	Economic institutional environment	Marketization process	The relationship between government and market (*X*_*10*_)	Ascending type
			The development of non-state-owned economy (*X*_*11*_)	Ascending type
			Market development degree (*X*_*12*_)	Ascending type
			Factor market development degree (*X*_*13*_)	Ascending type
			The development of market intermediary organizations (*X*_*14*_)	Ascending type

### Calculation Method

For the evaluation of comprehensive indicators, the previous studies mostly established the evaluation index system and used the analytic hierarchy process (AHP), multivariate statistical analysis, the Delphi method, and the entropy method to establish the evaluation function. However, these evaluation methods lack the dynamic consideration of “time dimension,” and even have serious random and speculative defects. Given this, in this article, the fully arranged polygon graphic indicator method is used, which has both static indicators and dynamic trends. It not only reflects the principle of system integration but also avoids the problem of overlapping information among multi-indicator variables and realizes a comprehensive review of the development of institutional quality in various provinces and cities in China from a dynamic point of view. The basic principle of the evaluation method is as follows: set *n* indicators, construct with the maximum value of these indexes as the radius (*n*–1)!/2 irregular central n-triangles, the vertices of which are the full arrangement of *n* indicators end to end. The composite index is the ratio of the average of all irregular polygon areas to the central polygon area. The specific calculation process is as follows:

(1) Building a standardized function:


(1) $$F\,\left(x\right)=\frac{a}{b\,x\,c}$$

In which, a, b, and c, respectively, represent the parameters of the hyperbolic function.

(2) The hyperbolic normalization function *F*(*x*) satisfies the following conditions: *F*(*U*) = 1, *F*(*T*) = 0, *F*(*L*) = –1, where u is the upper limit of index X, l is the lower limit of index X, t is the critical value of index X, and the critical value can be expressed by the average value of index X. Available from the above conditions:


(2) $$F\,\left(x\right)=\frac{\left(U-l\right)\,\left(x-T\right)}{\left(U+L-2\,T\right)\,x+U\,T+L\,T-2\,U\,T}$$

It can be seen from formula (2) that the standardization function *F*(*x*) maps the index value located in [L, U] to [−1, 1], and the standardization process will cause the index value to show a fast-slow-fast nonlinear growth trend.

(3) For the *i*th index, the standardized formula is expressed as follows:


(3) $$S_{i}\,\left(x\right)=\frac{\left(U_{i}-I_{i}\right)\,\left(x_{i}-T_{i}\right)}{\left(U_{i}+L_{i}-2\,T_{i}\right)\,x+U_{i}\,T_{i}+L_{i}\,T_{i}-2\,U\,T}$$

The vertex of the *n*-polygon is composed of *S_i_* = 1, and the center point consists of *S_i_* = –1, *S_i_* = 0 constitutes the critical value of the polygon index. If above the critical value, each index value is positive, and below the index value, each index value is negative.

(4) The comprehensive indexes of fully arranged polygons are as follows:


(4) $$S\,\left(x\right)=\frac{\sum_{i\neq j}^{i,j}\left(S_{i}+1\right)\,\left(S_{j}+1\right)}{2\,n\,\left(n-1\right)}$$

Among them, *S* is a comprehensive index and *S_i_* is a single indicator.

### Result Analysis

According to the results in Table 2, the average annual score of China’s institutional quality from 2010 to 2019 is 0.222. Except for the eastern and northeastern regions, the average annual institutional quality is higher than the national average, and all other regions are lower than the national average. The development ladder pattern of the eastern, northeastern, central, and western regions is obvious, and the ranking of regional institutional quality score is unchanged. The score of the new urbanization level in each province shows that except Hebei and Hainan, the average annual system quality scores in the eastern region are higher than the national average, while the average annual system quality scores in all provinces in the northeast region are not lower than the national average^1^. Only Henan in the central region is higher than the national average, while Inner Mongolia, Chongqing, and Ningxia in the western region are higher than the national average. Among them, the top 10 provinces with annual average system quality scores, 8 provinces (Beijing, Tianjin, Shanghai, Zhejiang, Jiangsu, Guangdong, Shandong, and Fujian) are from the eastern region, and 2 provinces (Liaoning and Jilin) are from the northeast region. Among the last ten provinces in terms of annual institutional quality, two provinces (Anhui and Jiangxi) are from the central region. Eight (Guangxi, Sichuan, Guizhou, Yunnan, Shaanxi, Gansu, Qinghai, and Xinjiang) are from the western region, and the calculation results basically accord with the current situation of China’s regional, political, and economic development. Table 2 shows the score and ranking of China’s regional institutional quality measurement. Due to space constraints, this article only lists the measurement results of some years.

**TABLE 2:** System quality measurement in some years in China from 2010 to 2019.

Province	2010		2013		2016		2019		Annual mean	
	Score	Ranking	Score	Ranking	Score	Ranking	Score	Ranking	Comprehensive score	Ranking
Beijing	0.279	3	0.332	3	0.421	2	0.463	4	0.383	3
Tianjin	0.281	2	0.381	1	0.434	1	0.427	10	0.395	1
Hebei	0.148	10	0.082	27	0.236	16	0.306	18	0.178	18
Shanghai	0.318	1	0.281	5	0.335	6	0.434	9	0.348	5
Jiangsu	0.177	8	0.235	7	0.281	10	0.434	8	0.285	9
Zhejiang	0.276	4	0.374	2	0.405	3	0.580	1	0.393	2
Fujian	0.200	7	0.262	6	0.332	7	0.449	7	0.312	6
Shandong	0.213	5	0.232	8	0.302	8	0.424	11	0.286	8
Guangdong	0.168	9	0.195	10	0.263	14	0.454	6	0.269	10
Hainan	0.076	24	0.134	19	0.192	19	0.247	24	0.158	20
Shanxi	0.121	15	0.178	13	0.232	17	0.333	16	0.211	16
Anhui (Province)	0.080	22	0.107	22	0.179	23	0.277	19	0.156	22
Jiangxi	0.076	23	0.102	24	0.162	25	0.270	21	0.150	24
Henan	0.133	13	0.193	11	0.274	12	0.363	14	0.232	13
Hubei	0.104	17	0.154	17	0.228	18	0.381	13	0.211	17
Hunan	0.106	16	0.146	18	0.182	22	0.219	26	0.158	19
Liaoning	0.203	6	0.296	4	0.358	4	0.540	2	0.361	4
Jilin	0.139	12	0.232	9	0.351	5	0.489	3	0.301	7
Amur	0.142	11	0.184	12	0.245	15	0.361	15	0.222	15
Inner Mongolia	0.097	19	0.168	15	0.264	13	0.460	5	0.242	11
Guangxi	0.071	25	0.091	25	0.144	26	0.219	27	0.130	26
Chongqing	0.124	14	0.173	14	0.275	11	0.325	17	0.228	14
Sichuan	0.090	20	0.102	23	0.167	24	0.261	23	0.154	23
Guizhou	0.029	28	0.059	28	0.100	29	0.164	29	0.086	29
Yunnan	0.016	30	0.088	26	0.186	20	0.261	22	0.126	27
Shaanxi	0.069	26	0.131	20	0.184	21	0.271	20	0.157	21
Gansu	0.033	27	0.056	29	0.118	28	0.199	28	0.099	28
Qinghai	0.028	29	0.050	30	0.094	30	0.152	30	0.076	30
Ningxia	0.088	21	0.165	16	0.282	9	0.385	12	0.232	12
Xinjiang	0.099	18	0.107	21	0.141	27	0.240	25	0.134	25
Eastern China	0.214	1	0.251	1	0.320	1	0.422	2	0.301	1
Middle China	0.104	4	0.147	4	0.209	4	0.307	4	0.186	4
Western China	0.068	5	0.108	5	0.178	5	0.267	5	0.151	5
Northeast China	0.161	2	0.237	2	0.318	2	0.463	1	0.295	2
National	0.133	3	0.176	3	0.246	3	0.346	3	0.222	3

## Model and Data

### Model Building

According to the research of Hao et al. (2021a), it is assumed that international technology spillover will affect the green innovation capability of the host country through FDI, OFDI, and foreign trade. Furthermore, the factors influencing the promotion of green innovation capability, such a human capital, R&D personnel investment, R&D capital investment, and industrial structure, are brought into the model. In addition, in this period, the regional innovation capability will be affected by the early stage, so the lag of innovation capability by one stage is added into the model as an explanatory variable, and the system generalized distance estimation (SYS-GMM) and differential generalized moment estimation (DIF-GMM) are used for estimation. Since the difference generalized moment estimation (DIFF-GMM) first removes the fixed effect of the model by difference, then, the lag period of explanatory variables is used as instrumental variables to construct difference equations, which can reduce the endogenous problems among variables, and the difficulty of searching instrumental variables (Irfan and Ahmad, 2021). The system GMM estimates the difference equation and the level equation as one equation, which can not only improve the efficiency of estimation but also estimate the coefficients of the variables that do not change with time in the model. So that the estimation result is more accurate. Therefore, in this article, the system GMM estimation results shall prevail in the concrete analysis, and the DIF-GMM estimation results are only for comparison without specific explanation. The benchmark model is set as follows:


$$l\,n\,c\,r\,e\,a\,t\,e_{i\,t}=\beta_{0}+\beta_{1}\,l\,n\,c\,r\,e\,a\,t\,e_{i\,t-1}+\beta_{2}\,l\,n\,f\,d\,i_{i\,t}$$

(5) $$+\gamma \,l\,n\,c\,o\,n\,t\,r\,o\,l_{i\,t}+\alpha_{i}+\varepsilon_{i\,t}$$

$$l\,n\,c\,r\,e\,a\,t\,e_{i\,t}=\beta_{0}+\beta_{1}\,l\,n\,c\,r\,e\,a\,t\,e_{i\,t-1}+\beta_{2}\,l\,n\,o\,f\,d\,i_{i\,t}$$

(6) $$+\gamma \,l\,n\,c\,o\,n\,t\,r\,o\,l_{i\,t}+\alpha_{i}+\varepsilon_{i\,t}$$

$$l\,n\,c\,r\,e\,a\,t\,e_{i\,t}=\beta_{0}+\beta_{1}\,l\,n\,c\,r\,e\,a\,t\,e_{i\,t-1}+\beta_{2}\,l\,n\,t\,r\,a\,d\,e_{i\,t}$$

(7) $$+\gamma \,l\,n\,c\,o\,n\,t\,r\,o\,l_{i\,t}+\alpha_{i}+\varepsilon_{i\,t}$$

To test the interactive effect (moderating effect) of institutional quality, this article introduces the interactive terms of institutional quality (inst), FDI, and foreign trade, respectively, and transforms the above equation into:


$$l\,n\,g\,m\,l_{i\,t}=\beta_{0}+\beta_{1}\,l\,n\,g\,m\,l_{i\,t-1}+\beta_{2}\,l\,n\,f\,d\,i_{i\,t}+\beta_{3}\,\left(i\,n\,s\,t_{i\,t}\times l\,n\,f\,d\,i_{i\,t}\right)$$

(8) $$+\gamma \,l\,n\,c\,o\,n\,t\,r\,o\,l_{i\,t}+\alpha_{i}+\varepsilon_{i\,t}$$

$$l\,n\,g\,m\,l_{i\,t}=\beta_{0}+\beta_{1}\,l\,n\,g\,m\,l_{i\,t-1}+\beta_{2}\,l\,n\,o\,f\,d\,i_{i\,t}$$

(9) $$+\beta_{3}\,\left(i\,n\,s\,t_{i\,t}\times l\,n\,o\,f\,d\,i_{i\,t}\right)+\gamma \,l\,n\,c\,o\,n\,t\,r\,o\,l_{i\,t}+\alpha_{i}+\varepsilon_{i\,t}$$

$$l\,n\,g\,m\,l_{i\,t}=\beta_{0}+\beta_{1}\,l\,n\,g\,m\,l_{i\,t-1}+\beta_{2}\,l\,n\,t\,r\,a\,d\,e_{i\,t}$$

(10) $$+\beta_{3}\,\left(i\,n\,s\,t_{i\,t}\times l\,n\,t\,r\,a\,d\,e_{i\,t}\right)+\gamma \,l\,n\,c\,o\,n\,t\,r\,o\,l_{i\,t}+\alpha_{i}+\varepsilon_{i\,t}$$

The interaction term is to preliminarily test the regulation effect of institutional quality by the exogenous grouping method. To avoid artificial division of growth intervals and estimation errors caused by endogenous problems in previous static threshold models, this article uses Wu et al. (2020) as a reference to study the dynamic threshold panel model and sets the following dynamic threshold panel model:


$$lncreate_{i\,t}=\beta_{0}+\beta_{1}lncreate_{i\,t-1}+\beta_{2}lnfdi_{i\,t}\cdot \text{I}\left(inst_{i\,t}\leq \text{c}\right)$$

(11) $$+\beta_{3}\,l\,n\,f\,d\,i_{i\,t}\cdot \text{I}\,i\,n\,s\,t_{i\,t}>\text{c}+\gamma \,l\,n\,c\,o\,n\,t\,r\,o\,l_{i\,t}+\alpha_{i}+\varepsilon_{i\,t}$$

$$lncreate_{i\,t}=\beta_{0}+\beta_{1}lncreate_{i\,t-1}+\beta_{2}lnofdi_{i\,t}\cdot \text{I}\left(inst_{i\,t}\leq \text{c}\right)$$

(12) $$+\beta_{3}\,l\,n\,o\,f\,d\,i_{i\,t}\cdot \text{I}\,i\,n\,s\,t_{i\,t}>\text{c}+\gamma \,l\,n\,c\,o\,n\,t\,r\,o\,l_{i\,t}+\alpha_{i}+\varepsilon_{i\,t}$$

$$lncreate_{i\,t}=\beta_{0}+\beta_{1}lncreate_{i\,t-1}+\beta_{2}lntrade_{i\,t}\cdot \text{I}\left(inst_{i\,t}\leq \text{c}\right)$$

(13) $$+\beta_{3}\,l\,n\,t\,r\,a\,d\,e_{i\,t}\cdot \text{I}\,i\,n\,s\,t_{i\,t}>\text{c}\,\gamma \,l\,n\,c\,o\,n\,t\,r\,o\,l_{i\,t}+\alpha_{i}+\varepsilon_{i\,t}$$

Among them, subscript I represents the province (*i* = 1,2,3…30), *t* represents the time, *create*_*it*_represents the green innovation ability, *create*_*it*−1_ a lagging term representing the green innovation ability, *fdi_it_* indicates FDI; *ofdi_it_* indicates OFDI; *trade_it_* represents foreign trade; *control*_*it*_ a series of control variables that affect the promotion of regional innovation capability, including the industrial structure adjustment index (*ind*_*it*_), R&D personnel investment (*rdp*_*it*_), R&D investment (*rd*_*it*_), human capital level (*hum*_*it*_); and *inst*_*it*_indicates the system quality, which is also a threshold variable; I(⋅) indicates the index function, and c is the specific threshold value;α_i_represents the individual fixation effect, in which α*_i_* = μ_*it*_ + υ_*it*_,μ*it* represents the regional fixed effect, _υit_ is the time fixed effect; and ε_*it*_ represents a random perturbation term.

### Explanation and Description of Variables

In this article, the number of green patent applications in different provinces is taken as the proxy variable of green innovation capability, and the stock of green innovation capability is calculated by the perpetual inventory method with reference to previous studies. Actual FDI, net non-financial FDI, and total import and export volume of China’s provinces over the years are used to represent FDI and foreign trade, respectively. The system quality shall be subject to the calculation results in Part II. With regard to control variables, the weighted average of the years of education of the population aged 6 years and above in each region is used to measure the human capital of each province, and the ratio of regional R&D investment to regional GDP is used to express the intensity of R&D investment, and the full-time equivalent of R&D personnel is used as the proxy variable of R&D personnel investment. The industrial structure adjustment index is expressed by the proportion of the annual output value of the tertiary industry and the annual output value of the secondary industry. Statistical information about each variable is shown in Table 3.

**TABLE 3:** Variable description and statistical description.

Variable name	Symbol	Unit	Calculation method
Green innovation ability	*gcreate*	piece	perpetual inventory system Calculated stock
Foreign direct investment (FDI)	*fdi*	Billion dollars	Taking 2006 as the base period Use directly after conversion.
FDI	*ofdi*	Billion dollars	Taking 2006 as the base period Use directly after conversion.
Foreign trade	*trade*	Billion dollars	Taking 2006 as the base period Use directly after conversion.
System quality	*inst*	−	Fully arranged polygon graph Indicator evaluation method
R&D personnel investment	*rdp*	ten thousand people	Use directly
R&D investment	*rd*	%	Use directly
Manpower capital	*hum*	year	Weighted mean number of years of education for population aged 6 and above
Industrial structure adjustment index	*ind*	%	Annual output value of tertiary industry/annual output value of secondary industry

## Results and Analysis

As mentioned earlier, this article focuses on the relationship between the three international technology spillovers of FDI, foreign trade, and China’s green innovation capability, and through what channels it influences China’s green innovation capability. Therefore, in the first section below, the direct effects of FDI and foreign trade on China’s regional innovation capability are tested, while in the second section, the interaction between institutional quality and three international technology spillovers is added to preliminarily test the regulatory effect of institutional quality. In the third section, the dynamic threshold panel model is introduced to further test the spillover effect of international technology under different institutional quality conditions.

### Direct Effect Analysis

Based on the panel data of 30 provinces in China from 2010 to 2019, the regression analysis of models (1) to (3) is carried out, and two-step SYS-GMM and two-step DIF-GMM are used to estimate the models, respectively. The results are shown in Table 4. It can be found that AR (2) test results show that there is no second-order sequence correlation in the random error term of the model, and Hansen test results show that the selection of model tool variables is effective. The Wald test results show that the overall height of the model is significant, so the regression results of SYS-GMM and DIF-GMM are reliable. At the same time, the direct effect estimation results also reflect the following problems.

**TABLE 4:** Direct effect estimation results.

Variable	Model 1		Model 2		Model 3	
	SYS-GMM	DIF-GMM	SYS-GMM	DIF-GMM	SYS-GMM	DIF-GMM
*lngcreate_*it*–1_*	0.708***	0.320***	0.559***	0.681***	0.883***	0.767***
	(76.23)	(2.63)	(11.21)	(34.61)	(69.96)	(11.18)
*lnrdp*	0.366***	2.544***	0.686***	0.675***	0.234***	0.764***
	(12.36)	(7.93)	(8.31)	(28.82)	(5.72)	(4.46)
*lnrd*	9.761***	−14.131*	40.055	−0.445***	21.749***	4.431
	(2.91)	(−1.84)	(1.45)	(−2.70)	(4.20)	(1.56)
*lnhum*	0.093	−4.526***	−0.635	−2.171***	−0.556***	−1.581**
	(0.53)	(−3.41)	(−1.22)	(−6.56)	(−4.42)	(−2.41)
*lnind*	−9.529***	15.923*	−39.937	−0.445***	−21.726***	−6.098*
	(−2.86)	(1.95)	(−1.44)	(−2.70)	(−4.20)	(−1.89)
*lnfdi*	0.212***	0.383***				
	(15.89)	(2.63)				
*lnofdi*			0.157***	0.121***		
			(7.28)	(9.25)		
*lntrade*					0.039***	0.001
					(6.18)	(0.02)
*_cons*	0.934***		3.609***		2.048***	
	(2.62)		(3.72)		(8.85)	
*AR(2)*	1.54	1.14	−0.32	1.25	1.21	−1.36
	[0.123]	[0.255]	[0.752]	[0.211]	[0.228]	[0.173]
*Hansen Test*	29.36	13.69	25.3	25.84	27.71	22.55
	[0.966]	[0.396]	[0.151]	[0.309]	[0.149]	[0.126]
*Wald Test*	128516.67***	353.93***	6234.02***	709949.2***	104446.29***	5849.14***
*Obs*	270	240	270	240	270	240

[] Denotes the corresponding Z value and () represents the corresponding value of p. *p value < 0.10, **p value < 0.05, ***p value < 0.01.

Foreign direct investment and foreign trade have significantly promoted the improvement of China’s green innovation capability, and their coefficients are all significantly positive at least at the level of 1%. The reason is that compared with the local enterprises in the host country, FDI enterprises usually have certain ownership advantages, and FDI with advanced technology has the potential for technology spillover (Khachoo et al., 2018). This will produce positive external spillover effects in the host country in four ways: demonstration effect, competition effect, personnel flow, and industrial correlation effect, thus promoting the technological progress and efficiency of the host country’s enterprises. OFDI enterprises can learn from the leading technology of local enterprises and absorb the local technology spillover when making international investments abroad. The subsidiaries carry out local technological innovation and realize technological progress, and then use various ways to introduce technology to the home country to realize reverse technology spillover. However, foreign trade technology spillovers often acquire knowledge useful to our country through international trade, technology exchange, and other activities. This is a good way for developing countries and regions to gradually narrow the economic gap with developed countries (Wu et al., 2019). The larger the foreign trade volume, the more contacts among countries (regions). These contacts will promote the exchange of technical information among regions and help trade importing countries to get some new innovations from these technologies. It is beneficial for foreign demanders to put forward improvement suggestions on the production process of exported products to promote the improvement of domestic green innovation ability.

### Analysis of Interaction Effect

Two-step SYS-GMM and two-step DIF-GMM are used to estimate models (4)–(6) after the interaction term is added. Table 5 interaction effect estimation results show that there is no second-order sequence correlation in the residual series, tool variable selection is effective, and the model is significant as a whole. As for the regulation effect model of system quality, the interaction coefficient between the three kinds of international technology spillovers and various institutional quality is significantly positive, which indicates that institutional quality will affect the determinant coefficient of international technology spillover on China’s green innovation capability. That is, the higher the quality of China’s system, the more favorable it is for FDI and foreign trade technology spillover. The reasons are as follows: in terms of the regulatory effect of institutional quality on FDI, first, a good institutional environment improves the efficiency of capital allocation and reduces the entry cost of FDI, which is not only conducive to the entry of foreign capital in quantity but also conducive to the entry of technology-oriented FDI in quality, and promotes the transformation and upgrading of China’s foreign capital structure (Urban, 2010). In addition, regions with higher institutional quality create a good institutional environment for the emergence of the FDI technology spillover effect, and the emergence of the FDI technology spillover effect provides a possibility for the improvement of China’s green innovation capability (Hao et al., 2020). Second, the high-quality institutional environment has stimulated the vitality of the regional market to gain profits in the fierce market competition, local enterprises will continue to increase R&D investment and enhance green innovation ability. The improvement of the innovation ability of local enterprises provides the possibility of absorbing FDI technology spillovers. At the same time, a high-quality institutional environment is conducive to the flow of regional technical personnel and provides favorable opportunities for FDI enterprises to spread technology and local enterprises to imitate and innovate, thereby promoting green innovation ability. In terms of the regulatory effect of institutional quality on OFDI, first, the implementation of the strategy of “invigorating the country through science and education” and “strengthening the country with talents” has promoted the improvement of China’s innovation ability and potential, which not only lays the foundation for the emergence of technology-oriented OFDI but also provides rich human capital for the home country enterprises to absorb the OFDI reverse technology spillovers. Second, the regions with higher system quality have an efficient financial market and an open market environment, and the policy support of the “going out” strategy not only provides convenience for OFDI enterprises to finance and invest but also helps them to integrate into a global value chain, participate in international market competition, and create conditions for technology seeking OFDI enterprises to absorb foreign advanced technologies (Chu et al., 2018). Third, the regions with higher system quality have a perfect management system, which is not only conducive to the management of OFDI multinational enterprises and reducing their operating costs but also provides institutional support for the return of technical personnel of overseas subsidiaries of OFDI enterprises, and creates a good institutional environment for promoting the green innovation ability of home countries. As far as the regulatory effect of institutional quality on foreign trade is concerned, for a long time, China’s technological progress is dominated by technological innovation and technology introduction. High-quality intellectual property protection can prevent patent infringement. It can not only protect high-tech imported products but also promote the increase of their quantity to a certain extent. By learning and imitating imported products with advanced technology, Chinese enterprises can promote the production of new technologies and new processes and improve their technological innovation ability. At the same time, regions with a high level of intellectual property protection provide institutional support for technology-oriented export enterprises to obtain high export trade profits and encourage domestic enterprises to increase research and development and investment in high-tech products, to promote China’s green innovation ability.

**TABLE 5:** Regression results of interaction effects.

Variable	Model 4		Model 5		Model 6	
	SYS-GMM	DIF-GMM	SYS-GMM	DIF-GMM	SYS-GMM	DIF-GMM
*lngcreate_*it*–1_*	0.802***	0.400***	0.790***	0.444***	0.795***	0.576***
	(76.64)	(5.46)	(50.57)	(7.42)	(16.29)	(35.70)
*lnrdp*	0.328***	2.242***	0.349***	2.013***	0.361***	1.107***
	(14.81)	(11.48)	(19.66)	(12.44)	(5.44)	(47.65)
*lnrd*	18.438**	−59.742	16.267***	−69.096*	88.804*	1.426
	(2.17)	(−1.43)	(2.73)	(−1.93)	(1.95)	(0.24)
*lnhum*	−1.075***	−5.205***	−1.285***	−4.263***	−0.055	−3.712***
	(−5.71)	(−5.31)	(−7.12)	(−5.50)	(−0.13)	(−10.89)
*lnind*	−18.313**	59.545	−16.045***	68.620*	−88.700*	−2.003
	(−2.16)	(1.42)	(−2.70)	(1.90)	(−1.95)	(−0.34)
*lnfdi*	0.084***	0.130***				
	(3.79)	(1.88)				
*inst*×*lnfdi*	0.089***	0.290***				
	(3.27)	(3.62)				
*lnofdi*			0.133***	0.138***		
			(3.07)	(2.00)		
*inst*×*lnofdi*			0.164***	0.141*		
			(4.20)	(1.89)		
*lntrade*					0.082***	0.466***
					(2.03)	(2.37)
*inst*×*lntrade*					0.198**	0.292***
					(2.39)	(11.26)
*_cons*	3.464***		4.016***		1.349*	
	(9.78)		(11.65)		(1.86)	
*AR(2)*	1.45	0.01	1.60	0.19	−0.27	0.96
	[0.147]	[0.992]	[0.11]	[0.848]	[0.788]	[0.338]
*Hansen Test*	29.45	19.49	27.57	23.33	27.7	3.77
	[0.928]	[0.301]	[0.981]	[0.273]	[0.426]	[0.438]
*Wald Test*	118312.07***	997.17***	59061.49***	1980.62***	16983.97***	26723.52***
*Obs*	270	240	270	240	270	240

[] Denotes corresponding Z value and () represents corresponding value of p. *p value < 0.10, **p value < 0.05, ***p value < 0.01.

### Dynamic Threshold Effect Analysis

#### Threshold Effect Test and Threshold Value Determination

Using Stata15 and based on the dynamic threshold panel model Wald test self-sampling method (bootstrap), the significance test of threshold effect with FDI, OFDI, and foreign trade as the core explanatory variables is conducted under the assumption of no threshold effect. From Wald statistics and its *p*-value, we can see that the dynamic threshold models with three different international technology spillovers as the core explanatory variables all rejected the original hypothesis of no threshold effect at the significance level of 1% (as shown in Table 6). This shows that the impact of international technology spillovers on regional green innovation capability is nonlinear due to the difference in institutional quality among provinces and regions.

**TABLE 6:** Self-sampling test of a dynamic threshold effect.

Core explanatory variable	Model	Threshold value	Wald statistic	*P*-value	BS times	95% confidence interval	
FDI	SYS-GMM	0.326	16.008***	0.000	1000	0.058	0.442
	DIF-GMM	0.085	55.380***	0.000	1000	0.058	0.442
OFDI	SYS-GMM	0.357	36.560***	0.000	1000	0.058	0.442
	DIF-GMM	0.430	222.818***	0.000	1000	0.058	0.442
Trade	SYS-GMM	0.442	118.123***	0.000	1000	0.058	0.442
	DIF-GMM	0.085	1.130***	0.000	1000	0.058	0.442

***Significant at the level of 1. P-value and critical value are obtained by repeated sampling of the GMM threshold panel regression program for 1,000 times. Wald statistic is used to judge whether the threshold feature is obvious. The smaller the corresponding probability, the more obvious the threshold feature is.

#### Parameter Estimation and Result Analysis

The threshold effect estimation results show (Tables 6, 7) that the positive effects of three kinds of international technology spillovers on green innovation capability all increase with the improvement of China’s institutional quality. Therefore, the international technology spillover effect is more obvious in regions with high institutional quality, which is consistent with the previous conclusion of the interaction effect. Specifically, with FDI as the core explanatory variable, if the regional system quality is lower than the threshold value of 0.326, the green innovation ability will increase by 0.090% for every 1% increase in FDI, and 0.105% for every 1% increase in FDI when the regional system quality is higher than the threshold value of 0.326. For OFDI technology spillovers, if the regional institutional quality is lower than the threshold value of 0.357, the green innovation ability will increase by 0.046% for every 1% increase in OFDI, and if the regional institutional quality is higher than the threshold value of 0.357, the OFDI will increase by 1%. Then, the green innovation ability will be improved by 0.056%. For foreign trade technology spillover, if the regional system quality is lower than the threshold value of 0.442, there is no obvious technology spillover effect. When the regional system quality is higher than the threshold value of 0.442, the regional innovation ability will increase by 0.095% for every 1% increase in foreign trade. International technology spillovers from three different channels in areas with low system quality, FDI has the largest technology spillover effect, followed by OFDI. In regions with high institutional quality, the technology spillover effect of FDI is the largest, followed by that of foreign trade and OFDI.

**TABLE 7:** Dynamic threshold regression results.

Variable	Model (1)		Model (2)		Model (3)	
	SYS-GMM	DIF-GMM	SYS-GMM	DIF-GMM	SYS-GMM	DIF-GMM
*lngcreate_*it*–1_*	0.856***	0.358***	0.819***	0.476***	0.977***	0.605***
	(89.83)	(11.84)	(87.54)	(39.86)	(50.62)	(4.02)
*lnrdp*	0.185***	1.645***	0.208***	0.727***	0.046	1.214***
	(19.12)	(20.31)	(13.69)	(21.91)	(0.84)	(5.51)
*lnrd*	−0.290***	0.183**	0.187***	0.028***	0.105	−0.015
	(−1.78)	(2.16)	(7.37)	(3.13)	(1.19)	(−0.48)
*lnhum*	−1.466***	−2.388***	−0.619***	−0.055	−2.751***	−6.704***
	(−6.16)	(−5.17)	(−3.96)	(−0.21)	(−5.80)	(−3.74)
*lnind*	−0.290*	−2.685***	0.187***	−1.018***	0.005	4.314**
	(−1.78)	(−11.92)	(7.37)	(−5.43)	(0.03)	(2.44)
*lnfdi*⋅*I*(*inst*≤*C*)	0.090***	0.233***				
	(12.01)	(9.22)				
*lnfdi*⋅*I*(*inst*≥*C*)	0.105***	0.919***				
	(13.76)	(11.26)				
*lnofdi*⋅*I*(*inst*≤*C*)			0.046***	0.115***		
			(4.43)	(8.76)		
*lnofdi*⋅*I*(*inst*≥*C*)			0.056***	0.165***		
			(8.44)	(10.16)		
*lntrade*⋅*I*(*inst*≤*C*)					0.076	0.747***
					(1.59)	(4.05)
*lntrade*⋅*I*(*inst*≥*C*)					0.095*	0.797**
					(1.86)	(3.66)
*_cons*	4.018***		2.637***		5.981***	
	(8.76)		(8.22)		(7.00)	
*AR(2)*	1.05	1.44	1.43	1.57	1.43	1.65
	[0.294]	[1.149]	[0.153]	[0.117]	[0.153]	[0.099]
*Hansen Test*	27.91	28.16	28.6	27.47	27.76	7.16
	[0.979]	[0.852]	[0.955]	[0.814]	[0.583]	[0.711]
*Wald Test*	76526.19***	6298.16***	103958.31***	25143.82***	50292.64***	605.69***
*Obs*	270	240	270	240	270	240

[] Indicates the corresponding Z value and () indicates the corresponding value of p. *p value < 0.10, **p value < 0.05, ***p value < 0.01.

## Conclusion and Policy Recommendation

In this article, the provincial panel data of China from 2010 to 2019 are used to measure the quality of China’s provincial system, and the system quality evaluation system is constructed by the method of fully arranged polygon graphic indicators, which is used as the adjustment variable to join the model. A dynamic panel model and a dynamic threshold panel model are used to test the direct effect, system quality interaction effect, and threshold effect of FDI and foreign trade spillover on green innovation capability. The results show that the three technology spillovers have significantly promoted China’s green innovation capability. System quality will affect the determining coefficient of international technology spillovers on China’s green innovation capability. The positive promoting effects of FDI and foreign trade on China’s green innovation capability all increase with the improvement of China’s system quality. In view of the above conclusions to use international technology spillover to promote China’s green innovation capability, this article puts forward the following suggestions:

First, continuously increase infrastructure construction, improve laws and regulations, continue to expand investment attraction, and create a good institutional environment for the continuous entry of FDI and its technology spillover. In the process of introducing foreign capital, the government should change the evaluation standard of heroes based on quantity theory, establish a performance evaluation system based on technology-oriented FDI introduction, and gradually improve the quality of FDI introduction. Constantly deepen reform and opening up, market-oriented, stimulate market vitality, and force enterprises to carry out green innovation ability with highly active market competition environment. Attach great importance to education, improve the level of regional human capital, and promote the absorptive capacity of local enterprises to FDI spillover technology (Wang, 2007; Deng et al., 2018). Liberate and relax the system of human resource management, promote the free flow of technical personnel in enterprises, and give full play to the effect of personnel mobility to promote technology dissemination. Second, continue to implement the strategy of “rejuvenating the country through science and education” and “strengthening the country through talents,” increase investment in science and technology and education, promote the innovation ability of the home country, and create conditions for the generation of technical OFDI in the home country. Intensify the reform of the financial market, improve the efficiency of the financial market, and provide a good financing environment for OFDI enterprises. Increase investment in developed countries, encourage technology-seeking OFDI, focus on investment in high-tech industries, and further optimize OFDI investment structure. Promote enterprise management innovation, promote the management level of multinational companies, and create favorable conditions for OFDI enterprises to return overseas technicians. Third, continue to implement the basic national policy of “opening to the outside world.” Adhere to the combination of “bringing in” and “going out” to expand the import and export trade volume. Improve the intellectual property protection system, encourage technological innovation of local enterprises, give policy support to technology-oriented export enterprises, and reward the export of high-tech products. Increase the import proportion of technology-oriented products and encourage Chinese enterprises to digest, absorb, and re-innovate foreign advanced technologies. Broaden communication channels at home and abroad, take customer demand as the guide, and constantly improve the added value of export products.

Although this article studies the relationship between international technology spillovers, institutional quality, and green innovation, provincial panel data are used as research samples. Future research may need to use urban data or enterprise data to get more accurate results.

## Data Availability Statement

The original contributions presented in the study are included in the article/supplementary material, further inquiries can be directed to the corresponding author/s.

## Author Contributions

TW contributed to conceptualization, writing—original draft, and methodology. YD contributed to supervision. KG contributed to formal analysis. RS contributed to variable construction. CW contributed to funding acquisition. BY contributed to data handling. All authors have read and agreed to the published version of the manuscript.

## Conflict of Interest

The authors declare that the research was conducted in the absence of any commercial or financial relationships that could be construed as a potential conflict of interest.

## Publisher’s Note

All claims expressed in this article are solely those of the authors and do not necessarily represent those of their affiliated organizations, or those of the publisher, the editors and the reviewers. Any product that may be evaluated in this article, or claim that may be made by its manufacturer, is not guaranteed or endorsed by the publisher.

## Footnotes

1 For the convenience of analysis, the term “province” is utilized to represent all provincial administrative units in China, such as provinces, municipalities, and minority autonomous regions.
